# Investigating the Effects of Dapagliflozin on Cardiac Function, Inflammatory Response, and Cardiovascular Outcome in Patients with STEMI Complicated with T2DM after PCI

**DOI:** 10.1155/2021/9388562

**Published:** 2021-10-15

**Authors:** LiMing Xue, Xian Yuan, Shuguang Zhang, Xia Zhao

**Affiliations:** ^1^Department of Cardiology, Lianshui County People's Hospital, Huaian, Jiangsu 223400, China; ^2^Department of Cardiology, The Second People's Hospital of Huai'an, Huai'an Hospital Affiliated to Xuzhou Medical University, Huaian, Jiangsu 223002, China; ^3^Department of Cardiology, Huai'an TCM Hospital Affiliated to Nanjing University of Traditional Chinese Medicine, Huaian, Jiangsu 223001, China; ^4^Department of Cardiology, The Second Affiliated Hospital of Jiaxing University, Jiaxing, Zhejiang 314000, China

## Abstract

**Objective:**

To explore the effect of dapagliflozin on cardiac function, inflammation, and cardiovascular outcome in patients with ST-segment elevation myocardial infarction (STEMI) combined with type 2 diabetes (T2DM) after percutaneous coronary intervention (PCI).

**Methods:**

70 patients with STEMI and T2DM were divided into the control group (*n* = 35) and the observation group (*n* = 35). Before surgery, patients in both groups were given conventional treatments such as coronary expansion, antiplatelet, anticoagulation, and thrombolysis, and PCI was performed. After the operation, both groups were given conventional antiplatelet, anticoagulation, lipid-lowering, and hypoglycemic treatments. On this basis, the observation group was treated with dapagliflozin tablets for 24 weeks. We observe and compare the left ventricular end-diastolic diameter (LVEDD), left ventricular end-systolic diameter (LVESD) and left ventricular ejection fraction (LVEF), myocardial enzyme spectrum, inflammatory reaction, and occurrence of adverse cardiovascular events (MACE) of the two groups of patients before and after treatment.

**Results:**

After treatment, the LVEDD and LVESD of the two groups were lower than those before treatment, and the observation group was lower than the control group (*P* < 0.05). The LVEF of both groups was higher than that before treatment, and the observation group was higher than the control group (*P* < 0.05). After treatment, the levels of two groups' patients' creatine kinase (CK), creatine kinase isoenzyme (CK-MB), and troponin I (cTnI) were all lower than those before treatment, and the observation group patients were all lower than the control group (*P* < 0.05). After treatment, the levels of serum myeloperoxidase (MPO), C-reactive protein (CRP), interleukin 6 (IL-6), and tumor necrosis factor-*α* (TNF-*α*) in the two groups were all lower than those before treatment, and the observation group patients were all lower than the control group (*P* < 0.05). After treatment, there was no statistical difference between the two groups of patients in cardiogenic death, recurrent myocardial infarction, and other adverse cardiovascular events (*P* > 0.05). But, the incidence of severe arrhythmia and heart failure in the observation group were both lower than those in the control group (*P* < 0.05). Kaplan–Meier survival curve analysis showed that the median survival time without MACE in the observation group was higher than that in the control group (*P* < 0.05).

**Conclusion:**

Dapagliflozin treatment for patients with STEMI combined with T2DM after PCI can improve cardiac function to certain extent, reduce inflammation, and will reduce the incidence of adverse cardiovascular outcomes.

## 1. Introduction

ST-segment elevation myocardial infarction (STEMI) refers to coronary atherosclerosis that forms thrombosis and causes lumen obstruction, which causes acute and persistent coronary artery ischemia and hypoxia. It often manifests as severe pain in the precordial area for more than 30 minutes and a sense of dying, and the ST segment of the electrocardiogram is obviously elevated [1]. Type 2 diabetes mellitus (T2DM) with long-term poor blood glucose control in patients is one of the important risk factors for STEMI [2, 3]. Opening the infarct-related arteries as soon as possible is the key to the treatment of STEMI patients. In STEMI patients with T2DM, the coronary arteries are characterized by multiple and diffuse lesions, and the coronary microcirculation is also damaged to varying degrees. The narrow range of myocardial arteries is wide, and it is difficult to form collateral circulation. Once MI occurs, its infarct size is larger; at the same time, the long-term hyperglycemia state causes an increase in the effective circulating blood volume, aggravates the heart load, easily causes heart failure, increases the mortality rate, and seriously affects the prognosis. At present, the basic principle and best strategy of STEMI treatment is to dredge the responsible blood vessel-reperfusion as early as possible, adequately, and continuously. Drug thrombolytic therapy can greatly increase the risk of important organ bleeding in STEMI patients with T2DM, and percutaneous coronary intervention (PCI) can quickly recanalize infarct-related artery (IRA) and restore myocardial blood supply that it is an effective method to efficiently save the dying myocardium in patients with STEMI and T2DM and has important clinical significance for restoring the patient's left heart function and reducing the occurrence of heart failure. PCI is also currently a common clinical treatment for STEMI.

In recent years, our country's medical emergency system has been continuously improved, especially the establishment of the chest pain center, which enables STEMI patients to receive timely intervention and greatly improves the patient's prognosis. However, in clinical practice, due to the lack of understanding of the disease in some patients with STEMI and T2DM, the atypical symptoms of precordial squeezing pain, the relatively late consultation time, and the refusal of interventional therapy by patients and their families, these patients missed the opportunity to open as soon as possible. IRA restores the chance of myocardial reperfusion, and a series of fatal complications occur, which seriously affect the health of patients. For STEMI patients with T2DM, due to long-term hyperglycemia, oxidative stress, etc., the inflammatory response after PCI is enhanced, and the incidence of adverse cardiovascular outcomes is significantly increased [4]. Therefore, for STEMI patients with T2DM after PCI, it is particularly important to actively control blood glucose and improve cardiovascular benefits. Dapagliflozin can reduce the reabsorption of urine glucose by inhibiting sodium-glucose cotransporter 2 (SGLT2), thereby lowering blood sugar levels [5]. In addition to lowering blood sugar, dapagliflozin also has cardiovascular protection and reduces the mortality rate of cardiovascular diseases [6]. In this study, patients with STEMI and T2DM were treated with dapagliflozin after PCI to observe its effect on inflammation and cardiovascular outcomes. The specific reports are as follows.

## 2. Materials and Methods

### 2.1. General Information

A total of 70 STEMI patients with T2DM who were admitted to four hospitals from September 2018 to October 2019 were selected, including 41 males and 29 females, and divided into the control group and the observation group, with 35 cases in each group as shown in Table 1. All patients met the diagnostic criteria for STEMI combined with T2DM [7, 8] and underwent PCI surgery. Those who are allergic to experimental drugs, patients who have received SGLT2 drug treatment, patients with severe liver and kidney dysfunction, and patients with other serious diseases were excluded. This study was approved by the ethics committee of our hospital, and all patients and their families signed an informed consent form.

### 2.2. Research Methods

All patients were given ECG monitoring, oxygen inhalation, coronary dilatation, antiplatelet, anticoagulation, and thrombolysis. PCI was performed within 12 hours after the patient's onset. The radial artery was routinely punctured, and coronary angiography was performed to determine the location of the infarct-related arterial disease. The stent was inserted to complete the PCI treatment. After the operation, they were given conventional antiplatelet, anticoagulation, lipid regulation, plaque stabilization, and blood sugar control treatments. On this basis, the observation group were given dapagliflozin tablets (AstraZeneca Pharmaceutical Co., Ltd., National Medicine Standard: J20170040) orally, 5 mg/d in the first week, and 10 mg/d thereafter and took it after meals, once in the morning and once in the evening. Both groups of patients were treated continuously for 24 weeks.

### 2.3. Observation Indicators

#### 2.3.1. General Information

It included two groups of patients' age, gender, body mass index (BMI), duration of diabetes, systolic blood pressure, diastolic blood pressure, smoking, Gensini score [9], history of hypertension, history of myocardial infarction, history of atrial fibrillation, history of stroke, and peripheral artery medical history.

#### 2.3.2. Hemodynamic Parameters

A cardiac color Doppler ultrasound was used to detect the left ventricular end-diastolic diameter (LVEDD), left ventricular end-systolic diameter (LVESD), and left ventricular ejection fraction (LVEF) before and after treatment.

#### 2.3.3. Myocardial Enzymes

The fasting venous blood of the two groups of patients before and after treatment was collected, placed in an anticoagulation tube, and centrifuged for 5 min in an 8 cm centrifuge at 1000 rpm, and the supernatant was collected and stored at −20°C for testing. Immunofluorescence was used to detect creatine kinase (CK), creatine kinase isoenzyme (CK-MB), and troponin I (cTnI) in the two groups before and after treatment.

#### 2.3.4. Inflammation

Enzyme-linked immunosorbent assay (ELISA) was used to detect serum myeloperoxidase (MPO), C-reactive protein (CRP), interleukin 6 (IL-6), and tumor necrosis factor-*α* (TNF-*α*) before and after treatment in the two groups level.

#### 2.3.5. Cardiovascular Outcomes

The occurrence of adverse cardiovascular events (MACE) during the treatment period was observed, including cardiogenic death, recurrent myocardial infarction, severe arrhythmia, heart failure, and other cardiovascular adverse events. The 12-month prognosis of MACE was observed. Both groups of patients were followed up for 12 months, with MACE as the end point, and the occurrence of MACE events in the patients was statistically analysed.

### 2.4. Statistical Methods

SPSS 22.0 software was used for processing, measurement data were expressed as mean ± standard deviation ($\bar{x}$ ±*s*), the *t*-test was used for comparison, count data were expressed by (%), and the *χ*^2^ test was used for comparison. The Kaplan–Meier survival curve was used to fit the occurrence of MACE events. The log-rank test was used to compare the incidence of MACE between the two groups. *P* < 0.05 indicated that the difference was statistically significant.

## 3. Results

### 3.1. Comparison of General Information of the Two Groups of Patients

General data such as age, gender, BMI, diabetes duration, systolic blood pressure, diastolic blood pressure, smoking, Gensini score, history of hypertension, history of myocardial infarction, history of atrial fibrillation, history of stroke, and history of peripheral artery disease were balanced and comparable in the two groups. The difference was not statistically significant (*P* > 0.05), as shown in Table 1.

### 3.2. Comparison of Hemodynamic Parameters of the Two Groups of Patients before and after Treatment

After treatment, the LVEDD and LVESD of the two groups of patients were lower than before treatment, the observation group was lower than the control group, and the difference was statistically significant (*P* < 0.05); after treatment, the LVEF of both groups was higher than that before treatment, the observation group was higher than the control group, and the difference were statistically significant (*P* < 0.05), as shown in Table 2.

### 3.3. Comparison of Myocardial Enzymes before and after Treatment in the Two Groups

After treatment, the serum CK, CK-MB, and cTnI levels of the two groups of patients were lower than those before treatment, and the observation group was lower than the control group. The differences were statistically significant (*P* < 0.05), as shown in Table 3.

### 3.4. Comparison of Inflammatory Response Levels between the Two Groups of Patients before and after Treatment

After treatment, the serum MPO, CRP, IL-6, and TNF-*α* levels of the two groups of patients were lower than those before treatment, and the observation group was lower than the control group. The differences were statistically significant (*P* < 0.05), as shown in Table 4.

### 3.5. Comparison of the Cardiovascular Outcomes of the Two Groups of Patients

After treatment, there was no statistical difference between the two groups of patients with cardiogenic death, recurrent myocardial infarction, and other adverse cardiovascular events (*P* > 0.05), but the incidence of severe arrhythmia and heart failure in the observation group was lower than that in the control group, and the difference was statistically significant (*P* < 0.05), as shown in Table 5. Kaplan–Meier survival curve results showed that the median survival time without MACE in the control group was 6 months, the median survival time without MACE in the observation group was 8 months, and the median survival time without MACE in the observation group was higher than that in the control group. The log-rank test was *P* = 0.002, as shown in Figure 1.

## 4. Discussion

With the continuous improvement of human living standards, the population of obesity and metabolic syndrome is increasing year by year, and the incidence of AMI in our country is showing an upward trend. STEMI is mainly caused by vascular blockage on the basis of coronary atherosclerosis, causing continuous reduction or interruption of IRA blood flow, resulting in insufficient myocardial oxygen supply. Ischemic myocardial infarction is characterized by loss of local myocardial systolic function, relatively increased pressure load in myocardial infarction area, decreased movement coordination of the entire left ventricular contractile wall, and left ventricular pressure overload, resulting in left ventricular dilation and morphological and structural changes, and ultimately affecting myocardial diastolic function, resulting in reduced left ventricular function. At the same time, myocardial ischemic changes tend to activate the sympathetic nervous system, renin-angiotensin-aldosterone system (RAAS), which makes the body produce a large number of endocrine hormones and accelerate the process of heart failure. Therefore, the fundamental measure to prevent heart failure after STEMI is to actively rescue the dying myocardium. Especially for T2DM patients with ST segment elevation myocardial infarction, coronary artery diffuses change, at the same time, long-term high blood sugar can make effective circulating blood volume increase, greatly increased cardiac preload and myocardial necrosis, more serious impact on cardiac function, easy to cause heart pump function obstacle, and a significant increase in the incidence and mortality of chronic congestive heart failure. In view of this, reducing heart failure in STEMI patients with DM has become the focus and difficulty of clinical research.

STEMI has a rapid-onset, extremely rapid disease progression and high mortality. It requires timely reperfusion therapy to dredge the occluded blood vessels [10–12]. PCI treatment of acute STEMI has the advantages of less trauma and fast postoperative recovery. It can effectively unblock the occluded infarcted blood vessel, realize coronary reperfusion, and restore the infarcted myocardium to the greatest extent. The incidence of myocardial infarction in T2DM patients is much higher than that in nondiabetic patients. Once STEMI occurs in patients with T2DM, continuous hyperglycemia and oxidative stress can aggravate the inflammatory response state, thereby increasing the incidence of MACE after PCI [13]. Therefore, for patients with STEMI combined with T2DM undergoing PCI after PCI, hypoglycemic drugs should be actively intervened to control blood sugar while minimizing the occurrence of MACE after surgery.

SGLT2 is a sodium-glucose cotransporter, which is distributed in the kidney and has a glucose reabsorption effect. Dapagliflozin is an SGLT2 inhibitor. Through a non-insulin-dependent mechanism, it inhibits the reabsorption of glucose in the kidney and can reduce the blood glucose concentration through the direct excretion of sugar in the urine. In the DECLARE-TIMI 58 cardiovascular prognosis study [14], it was pointed out that, in addition, to the hypoglycemic effect of dapagliflozin, it also has renal and cardiovascular protective effects. In this study, the LVEDD and LVESD of the two groups of patients were lower than those before treatment, and the LVEF was higher than that before treatment. Also, the observation group had lower LVEDD and LVESD than the control group, and LVEF was higher than that of the control group. Serum CK, CK-MB, and cTnI levels of the two groups of patients after treatment were lower than those before treatment, and the observation group was lower than the control group, suggesting that dapagliflozin has a certain protective effect on the heart function of STEMI patients with T2DM and can effectively restore the heart contraction function reduceing myocardial damage [15].

PCI can effectively open and occlude blood vessels and reduce the area of myocardial infarction. However, during the process of cardiac coronary stent placement, the stent will damage the vessel wall, which will lead to inflammation and further thrombosis [16]. The long-term persistent hyperglycemia in patients with STEMI and T2DM can aggravate the inflammatory response state, which in turn leads to severe MACE and other complications [17, 18]. CRP, IL-6, and TNF-*α* are common inflammatory factors. The increase in their levels can directly reflect the inflammation in the body. MPO exists in neutrophils, and the increase in their levels can predict the risk of myocardial infarction. It can participate in the regulation of oxidative stress and inflammation [19, 20]. The results of this study showed that the levels of serum MPO, CRP, IL-6, and TNF-*α* in the two groups were lower than those before treatment, and the observation group was lower than the control group. Dapagliflozin can reduce the level of oxidative stress by reducing blood sugar levels in the body, thereby reducing inflammation.

In this study, it was also found that the incidence of severe arrhythmia and heart failure in the observation group was lower than that in the control group. Kaplan–Meier survival curve results showed that the median MACE-free survival time of the observation group was higher than that of the control group. This is basically consistent with the results of other studies of dapagliflozin for the treatment of myocardial infarction [21, 22]. The possible reason is that dapagliflozin can reduce myocardial oxidative stress, reduce inflammation, prevent macrophage infiltration, and have cardiovascular protection. The results show that although dapagliflozin cannot prevent the appearance of cardiovascular diseases, it can reduce the incidence of severe cardiovascular diseases.

In summary, dapagliflozin treatment of STEMI patients with T2DM after PCI can improve heart function, reduce myocardial damage, reduce inflammation, reduce the occurrence of MACE, and protect the cardiovascular system.

## Figures and Tables

**Figure 1:** Survival curve of the two groups of patients with MACE.

**Table 1:** General information comparison (*n*, %, $\bar{x}$ ± *s*).

Index	Control group (*n* = 35)	Observation group (*n* = 35)	t/*χ*^2^/*Z* value	*P* value
Age	56.26 ± 9.76	58.58 ± 10.17	0.974	0.334
Men/women	21/14	20/15	0.059	0.808
BMI (kg/m^2^)	25.95 ± 3.64	26.12 ± 3.21	0.207	0.836
Diabetes time (age)	8.37 ± 7.12	9.11 ± 6.07	0.468	0.641
Systolic blood pressure (mmHg)	131.08 ± 17.43	129.05 ± 15.26	0.518	0.606
Diastolic blood pressure (mmHg)	79.93 ± 8.61	80.13 ± 7.12	0.106	0.916
Smoking	8 (22.86)	5 (14.29)	0.850	0.356

Gensini score				
≤30 score	7 (20.00)	8 (22.86)	0.085	0.771
>30∼60 score	22 (62.86)	20 (57.14)	0.238	0.626
>60 score	6 (17.14)	7(20.00)	0.095	0.759
History of hypertension	21 (60.00)	20 (57.14)	0.059	0.808
Past history of myocardial infarction	3 (8.57)	4 (11.43)	0.159	0.690
History of atrial fibrillation	2 (5.71)	1 (2.86)	0.348	0.555
History of stroke	2 (5.71)	3 (8.57)	0.215	0.643
History of peripheral arterial disease	1 (2.86)	2 (5.71)	0.348	0.555

**Table 2:** Comparison of hemodynamic parameters before and after treatment (*n*, $\bar{x}$ ± *s*).

Index	Time	Control group (*n* = 35)	Observation group (*n* = 35)	*t* value	*P* value
LVEDD (mm)	Before therapy	53.38 ± 10.65	53.27 ± 11.03	0.042	0.966
	After treatment	47.53 ± 8.49^*∗*^	40.07 ± 9.68^*∗*^	3.428	0.001

LVESD (mm)	Before therapy	34.16 ± 5.98	33.95 ± 6.17	0.145	0.886
	After treatment	30.84 ± 6.60^*∗*^	27.24 ± 6.57^*∗*^	2.287	0.025

LVEF (%)	Before therapy	40.76 ± 7.25	41.13 ± 7.11	0.216	0.830
	After treatment	47.29 ± 7.34^*∗*^	52.03 ± 6.88^*∗*^	2.787	0.007

*Note.* Compared with the same group before treatment, ^*∗*^*P* < 0.05.

**Table 3:** Comparison of myocardial enzymes before and after treatment (*n*, $\bar{x}$ ± *s*).

Index	Time	Control group (*n* = 35)	Observation group (*n* = 35)	*t* value	*P* value
CK (U/L)	Before therapy	269.59 ± 65.17	267.17 ± 64.21	0.156	0.876
	After treatment	152.31 ± 16.72^*∗*^	90.81 ± 9.76^*∗*^	18.793	≤0.001

CK-MB (U/L)	Before therapy	55.83 ± 6.88	56.67 ± 6.25	0.535	0.595
	After treatment	27.06 ± 3.47^*∗*^	12.82 ± 1.22^*∗*^	22.904	≤0.001

cTnI (ug/L)	Before therapy	0.18 ± 0.03	0.17 ± 0.02	1.641	0.106
	After treatment	0.07 ± 0.02^*∗*^	0.02 ± 0.01^*∗*^	15.875	≤0.001

*Note.* Compared with the same group before treatment, ^*∗*^*P* < 0.05.

**Table 4:** Comparison of inflammatory response levels before and after treatment (*n*, $\bar{x}$±*s*).

Index	Time	Control group (*n* = 35)	Observation group (*n* = 35)	*t* value	*P* value
MPO (ng/ml)	Before therapy	28.13 ± 5.46	28.01 ± 5.68	0.090	0.929
	After treatment	19.93 ± 4.39^*∗*^	11.86 ± 4.69^*∗*^	7.867	≤0.001

CRP (ug/ml)	Before therapy	14.81 ± 3.25	14.93 ± 3.16	0.157	0.876
	After treatment	8.31 ± 2.78^*∗*^	4.39 ± 1.81^*∗*^	6.991	≤0.001

IL-6 (pg/ml)	Before therapy	17.63 ± 3.36	19.06 ± 3.74	1.683	0.097
	After treatment	12.77 ± 2.83^*∗*^	7.02 ± 2.93^*∗*^	8.351	≤0.001

TNF-*α* (pg/ml)	Before therapy	31.23 ± 5.83	32.44 ± 5.17	0.919	0.362
	After treatment	23.27 ± 5.42^*∗*^	14.06 ± 4.51^*∗*^	7.728	≤0.001

**Table 5:** Comparison of cardiovascular outcomes between the two groups of patients (*n*, %).

Index	Control group (*n* = 35)	Observation group (*n* = 35)	*χ* ^*2*^ value	*P* value
Cardiac death	2 (5.71)	0 (0.00)	2.059	0.151
Recurrent myocardial infarction	3 (8.57)	1 (2.86)	1.061	0.303
Severe arrhythmia	8 (22.56)	2 (5.71)	4.200	0.040
Heart failure	6 (17.14)	1 (2.86)	3.968	0.046
Other cardiovascular adverse events	4 (11.43)	3 (8.57)	0.159	0.690

## Data Availability

The data used and analyzed during the current study are available from the corresponding author on reasonable request.
